The article "Tanshinone Protects against Spinal Cord Ischemia-Reperfusion Injury by Inhibiting JNK Activity" was retracted in 2022. Reason: concerns about the peer review.

# Tanshinone Protects against Spinal Cord Ischemia-Reperfusion Injury by Inhibiting JNK Activity

**DOI:** 10.1155/2022/7619797

**Published:** 2022-05-11

**Authors:** Peng Zhang, Qingyu Zhang, Xiaoyang Liu, Tao Li, Shuai Wu, Yi Li, Zhensong Jiang

**Affiliations:** Department of Orthopaedics, Shandong Provincial Hospital Affiliated to Shandong First Medical University, Jinan 250014, Shandong, China

## Abstract

Spinal cord reperfusion injury as a secondary damage after primary spinal cord injury is an important factor causing nerve cell damage. In this study, we aim to investigate the effects and mechanisms of tanshinone (TAE) in the rabbit spinal cord during ischemia-reperfusion. New Zealand white rabbits were randomly divided into 3 groups: sham-operated group (5 rabbits), ischemia-reperfusion group (0.9% TAE was administered intraperitoneally 30 min before ischemia, and 4 groups of 5 rabbits each according to different time periods of reperfusion: group A reperfused for 0.5 h, group B reperfused for 2 h, group C reperfused for 8 h, and group *D* reperfused for 24 h), and TAE group (an ischemia-reperfused for 24 h). Group A was reperfused for 0.5 h, group B for 2 h, group C for 8 h, group *D* for 24 h, and group TAE (TAE was applied 30 min before ischemia reperfusion, grouped as ischemia-reperfusion group). The expression of JNK (c-Jun NH2-terminal Kinase) and phosphorylation-JNK (p-JNK) in spinal cord tissues of each group were detected by Western blot. Light and electron microscopy showed that early apoptosis started in group B in the ischemia-reperfusion group, while early apoptosis appeared only in group *D* in the tanshinone intervention group. Western blot showed that p-JNK expression started in group B in the ischemia-reperfusion group and gradually increased with the prolongation of ischemia time, while p-JNK expression only increased in group *D* in the tanshinone intervention group. In the tanshinone intervention group, p-JNK was activated only in group *D* and its activity was less than that in the ischemia-reperfusion group; the protein expression of JNK did not change significantly in both groups. Spinal cord ischemia-reperfusion can cause spinal cord injury by activating the signaling molecule JNK (MRPKs family), and early tanshinone intervention can partially inhibit this injury. Our finding provides a new idea and theoretical basis for clinical treatment of spinal cord ischemia-reperfusion injury.

## 1. Introduction

Spinal cord ischemic reperfusion injury (SCI) is a phenomenon in which the blood supply to the spinal cord is restored after the removal of some factors causing spinal cord ischemia, but the neurological function is not improved, but further aggravated by the original ischemic injury, and even irreversible delayed death of spinal cord neurons occurs. Spinal cord ischemia-reperfusion injury can cause quadriplegia, paraplegia, and even death [1]. The exact mechanism of spinal cord reperfusion neuronal injury is still inconclusive. JNK was first discovered in 1993 by Hibi et al. [2] and is an important member of the MAPK family, which belongs to the serine/threonine protein kinase pathway, and is involved in the development of many apoptotic cells and can be activated by various stress signals or inflammatory factors such as TNF*α*, FAS, and Ros [3–5]. Previous studies have shown that spinal cord ischemia-reperfusion injury induces apoptosis in neuronal cells by inducing the separation of 14-3-3 from ASK1, which leads to the activation of ASK1, and then activates its downstream signaling molecule JNK [6]. Tanshinone is a powerful antioxidant with its own free radical scavenging function and deacetylates upon entry into cells to produce cysteine, which promotes the synthesis of glutathione. The latter is the main force in the cellular fight against oxidative stress damage [7, 8].

In recent years, studies have suggested that apoptosis of neuronal cells is involved in the process of spinal cord ischemia-reperfusion injury. Tanshinone, a rosin alkane diterpenoid compound, is the main fat-soluble active component of *Salvia miltiorrhiza*, a traditional Chinese medicine, with antibacterial, antioxidant, anti-inflammatory and antitumor activities [9]. Tanshinone acts as an antioxidant by reducing oxidative stress by reacting with peroxides and inhibiting the production of reactive oxygen species (ROS) [10, 11]. Previous studies have shown that ROS are agonists of MAPK family members [12, 13]. Upstreams of JNK are at least two classes of kinases, MAPKKKs (ASK1) and MAPKKs (MKK4, MKK7), which sequentially phosphorylate and activate JNK through a cascade of reactions [14, 15]. Zhu et al. have demonstrated that tanshinone exerts its cerebral protective effects by scavenging reactive oxygen species (ROS) and inhibiting inflammatory responses during cerebral ischemia-reperfusion injury [16].

In this experiment, we investigated the effect of tanshinone on JNK activity in a rabbit spinal cord ischemia-reperfusion injury model, aiming to elucidate the protective mechanism of tanshinone against spinal cord ischemia-reperfusion injury.

## 2. Materials and Methods

### 2.1. Materials

Healthy male and female adult New Zealand rabbits (2-3 kg) were provided by the Animal Center of Nanjing Medical University; N-acetylcysteine was provided by Beyoncé Institute of Biotechnology (S0077); luminescence kits (cat# 7071), anti-JNK (cat# 9252), anti-phospho-JNK (cat# 9255) (Cell Signaling, USA). 9255) (Cell Signaling, USA).

### 2.2. Methodology

After intravenous anesthesia with 25% urutan (4 ml/kg) at the ear margins of healthy adult New Zealand rabbits, they were debrided, a median incision was made in the supine position, and the abdominal cavity was entered under aseptic conditions to locate the abdominal aorta, which was completely blocked by an arterial clip at the lower end of the renal artery [12]. After clamping the abdominal aorta for a predetermined time, the arterial clamp was released and the abdominal cavity was closed for reperfusion until a predetermined time. The animals were placed in the ventral recumbent position, the skin muscles of the back were incised, and the spinal canal was bitten open by biting forceps to expose the spinal cord, and the spinal cord below the L4 segment was taken. The spinal cord of normal animals was taken from the sham-operated group; the ischemia-reperfusion group was divided into four groups: 30 min ischemia/reperfusion for 0.5 h, 30 min ischemia/reperfusion for 2 h, 30 min ischemia/reperfusion for 8 h, and 30 min ischemia/reperfusion for 24 h. In each group, 5 ml of 0.9% tanshinone was administered 30 min before ischemia. The tanshinone intervention group was divided into 4 groups, the same as the ischemia-reperfusion group, and tanshinone 500 mg/kg (dissolved in 5 ml of 0.9% tanshinonel) was administered intraperitoneally 30 min before ischemia in each group.

The removed spinal cord tissue below the L4 segment was rapidly divided into 3 segments and fixed in 10% formaldehyde (for HE staining and immunohistochemistry), 5% glutaraldehyde (for electron microscopy), and stored at −70°C (for Western blot and immunoprecipitation), respectively. Spinal cord tissues stored at −70°C were lysed with tissue lysis solution [12] (50 mmol/L Tris (pH 7.4), 150 mmol/L tanshinonel, 1% NP-40, 0.25% sodium deoxycholate, 1 mmol/L EDTA, 1 mmol/L PMSF, 1 mmol/L PMSF, 1 mmol/L PMSF, 1 mmol/L PMSF, 1 mmol/L PMSF. mmol/L PMSF, 1 mmol/L aprotinin, 1 mmol/L Na3VO4) were lysed, the cell membranes were broken by ultrasound, the supernatant was centrifuged at 14 000 r/min for 10 min at 4°C, and the protein concentration was measured by BCA and then split and stored at −70°C.

Light microscopy sample preparation: Paraffin-embedded formalin-fixed spinal cord tissue, 4 *μ*m sections, fixed on poly-l-lysine-embedded slides for HE staining and light microscopy of the sections. Electron microscopy sample preparation: Spinal cord gray matter fixed with 5% glutaraldehyde was cut into 0.5 mm^3^ pieces, fixed with 5% glutaraldehyde for 2 hours at 4°C, and rinsed four times with phosphate buffer for 15 min each time. 1% osmium acid was fixed for 2 hours at 4°C and rinsed twice with a phosphate buffer for 5 min each time. 2% uranyl acetate aqueous solution was block-stained for 2 h and then dehydrated with 100% acetone: embedding agent (1 : 1) for 15 min at room temperature. After 2 h, the blocks were dehydrated at 4°C for 15 min with 50%, 70%, 90%, 100% and 100% acetone. The blocks were treated with 100% acetone: embedding agent (1 : 1) for 1.5 h at room temperature, 100% acetone: embedding agent (1 : 2) for 1.5 h at room temperature, and pure embedding agent for 3 h at 37°C. After embedding, the blocks were polymerized at 60°C for 36 h at room temperature. The nerve cells in the spinal cord tissue were observed by transmission electron microscopy after 36 h of polymerization at a constant temperature of 60°C.

The spinal cord tissue lysed by lysis solution was sampled with an equal amount of protein and then subjected to SDS gel electrophoresis and membrane transfer. The PVDF membrane was rinsed for 5 min at room temperature with 25 ml TBST. The blocking solution was blocked for 1 h at room temperature and rinsed 3 times for 5 min each with 15 ml TBST, anti-phospho-JNK 1 : 1 000, and anti-JNK 1 : 1 000. The PVDF membrane was incubated overnight at 4°C, in 15 ml TBST rinsed 3 times for 5 min each time. The PVDF membrane was incubated with secondary antibody (1 : 2 000) and anti-biotin antibody for marker detection (1 : 1 000) at 37 °C for 1 h rinsed with 15 ml TBST 3 times for 5 min each time. PVDF membranes were incubated with 1 ml of light-emitting solution (50 *μ*l 20 × LumiGLO, 50 *μ*l 20 × peroxide and 900 *μ*l Milli-Q water) for 1 min at room temperature, exposed in a dark room, developed and fixed.

Western blot films were scanned with a gel imaging system (UVP Company), and the grayscale values of the target bands were determined by Gel-Pro Analyzer software (Media Cybernetics). SPSS13.0 was used for statistical analysis, and the Student–Newman–Keuls method was used to compare the differences in protein expression between the experimental and control groups $\left(\bar{x}\pm s\right)$. In order to clarify the role and mechanism of tanshinone in spinal cord ischemia-reperfusion injury, the activation of JNK in specimens from the ischemia-reperfusion and tanshinone intervention groups was examined by Western blot.

## 3. Results

### 3.1. HE Staining and Electron Microscopic Observation

In the sham-operated group, the entire spinal cord tissue was intact and clear, with no obvious interstitial hemorrhage, normal nerve cell morphology, and clearly visible nuclei (Figure 1(a)). In the ischemia-reperfusion group, there was no significant change between groups A and B and the sham-operated group, while group C had a small amount of hemorrhage, mild swelling of nerve cells, and a mild decrease in nuclei (Figure 1(b)). In group *D*, the interstitial hemorrhage was significantly enlarged, and the nuclei of nerve cells were clearly visible (Figure 1(c)). There was a slight hemorrhage in the interstitium of spinal cord tissue, mild swelling of nerve cells, and a small decrease in nucleoli in group *D* (Figure 1(d)).

In the sham-operated group, the neuronal cell structure was clear and intact, the nuclear membrane was intact, and the nuclear chromatin was finely granular (Figure 2(a)). In the ischemia-reperfusion group, there was no significant change between group A and the sham-operated group. In the group B, the nuclear chromatin was borderline and condensed, the nuclear shape was irregular, the nucleolus was condensed, the cytoplasm was concentrated, and the number of vacuoles in the cytoplasm was increased (Figure 2(b)). In group *D*, the nucleus was fragmented, the nucleus was condensed, the nuclear chromatin was borderline and fragmented, the nuclear membrane was lost, and apoptotic vesicles were formed (Figure 2(c)). In the tanshinone intervention group, there were no significant changes in groups A, B, and C compared with the sham-operated group, while group *D* showed smaller cell size, increased vacuoles in the cytoplasm, uneven surface of the nuclear membrane, chromatin coalescence, crescentic shape of the inner nuclear border, disappearance of nuclear membrane pores, and corrugated and wrinkled nuclear membrane (Figure 2(d)).

### 3.2. Western Blot Detection of p-JNK and JNK Expression and Activation in the Spinal Cord Tissue

JNK expression was detected in the spinal cord tissue of all groups, and the expression amount did not differ significantly between groups (Figure 3(a)). The activation of JNK in the ischemia-reperfusion groups B, C, and *D* was significantly increased compared with the sham-operated group (*P* < 0.05), and the intensity of its expression increased with the increase of reperfusion time. The activation of JNK in the tanshinone intervention group *D* was increased compared with the sham-operated group (*P* < 0.05).

## 4. Discussions

Spinal cord reperfusion injury as a secondary damage after primary spinal cord injury is an important factor causing nerve cell damage, and the mechanism of injury is multifactorial, with possible mechanisms including ionic environment, oxygen-free radicals, and excitatory amino acids [17]. The MAPK signaling pathway exists in eukaryotic cells and is able to transduce different stimulatory signals from extracellular to nucleus, causing cell proliferation or apoptosis, and is widely used in the study of cell signaling. JNK was first discovered in 1993 by Hibi et al. [2] and is an important member of the MAPK family of serine/threonine protein kinase pathways, which have been shown to be involved in the development of apoptosis in many cells [2]. The JNK is activated by phosphorylation of its amino acid residues, and JNK is translocated to the nucleus upon activation. Previous studies have demonstrated that spinal cord ischemia-reperfusion injury can lead to apoptosis of spinal cord neuronal cells by inducing activation of ASK1, an upstream signaling molecule of JNK, which in turn activates JNK. Activated JNK mediates apoptosis mainly through two pathways: transcription-dependent and transcription-independent mechanisms. When acting through the transcription-dependent pathway, a portion of the active JNK moves to the nucleus to participate in gene transcription.

Compared with the tanshinone intervention group, the activation of JNK in the ischemia-reperfusion group started at 30 min/2 h of reperfusion and increased with the increase of reperfusion time, tanshinone where the activation of JNK started at 30 min/24 h of reperfusion. Levels in the tanshinone intervention group were lower than those in the ischemia-reperfusion group. The results showed that tanshinone preprotection significantly reduced JNK activation before spinal cord ischemia-reperfusion injury, probably because tanshinone, as a sulfhydryl reducing agent, could inhibit the separation of ASK1 and 14-3-3 by scavenging ROS and increasing GSH content in the body. The mechanism may be that tanshinone, as a sulfhydryl compound reducing agent, can inhibit the activation of JNK by scavenging ROS in vivo while increasing GSH content, inhibiting the separation of ASK1 and 14-3, thereby inhibiting the phosphorylation of ASK1, which in turn inhibits the activation of JNK in the transcriptional pathway, inhibiting apoptosis and protecting spinal cord tissue. Therefore, tanshinone not only has the effect of inhibiting oxidative stress but also directly inhibits the activation of JNK and directly inhibits apoptosis, which is consistent with the findings of Hui et al. and further explains the protective mechanism of tanshinone against neuronal cell injury [18].

## 5. Conclusion

In conclusion, this study found that tanshinone has the effect of inhibiting oxidative stress in spinal cord ischemia-reperfusion injury and can inhibit the activation of JNK and directly inhibit apoptosis. Meanwhile, tanshinone, as a commonly used drug, has the advantages of low price and clear side effects, which can generate great economic and social benefits if it can be widely used in the clinic to prevent spinal cord injury. However, JNK can also mediate apoptosis via a transcriptionally nondependent pathway, i.e., the mitochondrial pathway, and whether tanshinone affects this pathway needs further investigation.

## Figures and Tables

**Figure 1:** Morphological observations of the spinal cord (HE, × 400) (a) Spinal cord sections of the sham-operated group with normal nerve cell morphology and no interstitial hemorrhage; (b) spinal cord sections of the ischemia-reperfusion group with 30 min of ischemia/reperfusion for 2 h with mild swelling of nerve cells and a little interstitial hemorrhage; (c) spinal cord sections of the ischemia-reperfusion group with 30 min of ischemia/reperfusion for 24 h with significant swelling of nerve cells and significant interstitial lamellar hemorrhage; and (d) spinal cord sections from the tanshinone intervention group with 30 min of ischemia/reperfusion for 24 h with mild swelling of nerve cells and trace interstitial hemorrhage.

**Figure 2:** Observation of neurocytes morphology under electron microscope (a) Spinal cord cells in the sham-operated group with normal neuronal morphology (×10,000). (b) Spinal cord cells in the ischemia-reperfusion group with 30 min/reperfusion 2 h of ischemia, with chromatin-fragmented and condensed nuclei and concentrated cytoplasm (×20,000). (c) Spinal cord cells in the ischemia-reperfusion group, with nuclear fragmentation, loss of nuclear membrane, and formation of apoptotic vesicles (×20,000). (C) Spinal cord cells in the ischemia-reperfusion group, with nuclear fragmentation, loss of nuclear membrane, and formation of apoptotic vesicles (×20,000). (d) Spinal cord cells in the tanshinone intervention group with 30 min of ischemia/reperfusion for 24 h Nucleus consolidation and chromosome aggregation were slightly visible, and the nucleus also showed slight irregularity (×20,000).

**Figure 3:** Western blot detection of p-JNK and JNK expression in spinal cord tissue.

## Data Availability

The datasets used and/or analyzed during the current study are available from the corresponding author on reasonable request.
